# Knowledge Transfer Analysis and Management of Virtual Enterprises Based on Structured Cognitive Computing

**DOI:** 10.1155/2022/4858434

**Published:** 2022-02-22

**Authors:** Ai Lei

**Affiliations:** School of Information Management, Nanjing University, Nanjing 210023, China

## Abstract

With the advent of the era of big data, in the face of massive data mining, cognitive computing will play a pivotal role in future data processing. This study aims to study how to analyze the knowledge transfer and management of virtual enterprises based on structured cognitive computing. This study explains the basic concepts of structured cognitive computing and virtual enterprises and discusses knowledge transfer. In the experiment of this study, it can be seen from Table 1that in 2015, the growth rate of virtual enterprises reached 13%, the growth rate of virtual enterprises reached 36% in 2019, and it increased by 23% from 2015 to 2019. It can be seen that the development of virtual enterprises is getting faster and faster. From the data in Table 2 in the experiment of this study, we can see that with the increase in virtual enterprises in recent years, it has also brought development to the economy of various regions in China. The average employment rate in each region has increased by 24% at the lowest and reached 30% at the highest. It shows that the virtual enterprise has a great effect on the development of the region. Virtual enterprises can not only promote the growth of regional employment rate but also promote the flow of funds between different regions. Knowledge transfer is an important part of the sustainable development of virtual enterprises. How to carry out effective knowledge transfer and management has become a problem that contemporary virtual enterprises need to think about. There are three main factors that affect the knowledge transfer of virtual enterprises: knowledge transfer party, knowledge receiver, and virtual enterprise's own factors.

## 1. Introduction

Since the concept of the virtual enterprise was promoted, this business model has become more and more widely used in business. A virtual enterprise is a dynamic organization composed of multiple member companies promoted by related parties. From the moment the virtual enterprise was born, with its unique characteristics, it showed strong vitality and brought efficient benefits to the enterprise. With the rapid development of information technology, the business environment of enterprises has undergone great changes, and market competition has become increasingly fierce. Enterprises and organizations must respond to challenges and make decisions faster. Knowledge transfer and knowledge sharing have become the key to the success or failure of enterprises.

Different enterprise backgrounds make the entire virtual enterprise gather a lot of knowledge. Therefore, knowledge transfer provides a lot of resources, and the network organization structure of virtual enterprise provides a good platform for knowledge transfer. At the same time, the network organization structure of the virtual enterprise is very suitable for the flow of knowledge, so the related theoretical research is also enriched. Cognitive computing refers to intelligent systems that learn on a large scale, purposefully reason, and use natural language to interact with humans and other intelligent systems. These systems are not explicitly programmed but learn and reason from interaction. In the past half-century, developments in many scientific fields have enabled them to be realized.

The innovations of this study are as follows: (1) It introduces the relevant theoretical knowledge of cognitive computing and virtual enterprise knowledge transfer and uses the cloud model algorithm based on cognitive computing to analyze how structured cognitive computing is applied to virtual enterprise knowledge transfer. (2) Based on the cloud model algorithm and principal component analysis of cognitive computing, the experiment and analysis of the factors affecting the knowledge transfer of virtual enterprises are carried out. Finally, this study proposes how to carry out effective knowledge transfer measures according to the influencing factors of knowledge transfer.

## 2. Related Work

With the rapid development of virtual enterprises in recent years, the importance of knowledge transfer cannot be ignored. Giudice MD believes that people are living in a new era of economic development, the so-called era of knowledge economy, and knowledge seems to be the key foundation for value creation. In recent years, knowledge seems to have become an all-encompassing term. Therefore, he began to conduct research on the knowledge transfer of today's knowledge-intensive enterprises and found that knowledge transfer can promote the development of enterprises. His conclusion has not undergone any proof, and the authenticity is lacking [1]. Avventuroso et al. found that housing construction has always been organized and operated as a virtual enterprise. Choosing a suitable partner to establish a virtual enterprise is the key to implementing housing construction. He analyzed the connotation of virtual housing enterprises and established an index system based on the influencing factors of virtual enterprises. But he did not explain the specific role of this indicator system and how to establish this indicator system [2]. Nakayama et al. found that the sharing of tacit knowledge posed challenges. Traditional methods are prone to knowledge hoarding, and they are also prone to knowledge loss. Nakayama et al. proposed a model that can effectively solve the challenges brought about by the sharing of tacit knowledge and bring benefits to the storage of knowledge. However, the scholar did not conduct experiments on the model he proposed, so the reliability of the model has yet to be proven [3]. The purpose of Rupcic is to break through the challenges surrounding the process of learning and knowledge transfer and how to seize the opportunities brought by knowledge transfer. He discussed this aspect from the perspective of management and employees. He found that with the development of information and communication technology, knowledge transfer can be carried out by improving the learning agility of relevant personnel, thereby breaking through the challenges it brings. However, the scholar did not mention how to specifically break through the challenge [4]. Welch and Welch studied how multinational corporations develop their ability to operate in multiple languages to promote corporate communication, knowledge transfer, and absorptive capacity. Although the use of a common corporate language can play a huge role, it is difficult to meet the diverse foreign language needs that accompany global expansion by relying on this method alone. Therefore, relevant personnel should innovate their own knowledge to meet the needs of enterprises. The scholar's point of view is very good, but he did not propose a specific method of innovative knowledge transfer [5]. Bacon et al. believe that an open innovation ecosystem involves knowledge transfer among multiple stakeholders. It can promote the innovation of products and services and effectively manage the knowledge and information transferred between partners, which are essential for the open innovation process. He expanded existing knowledge by exploring the conditions for successful knowledge transfer between ecosystem partners and found that knowledge transfer is conducive to the self-improvement of partners. But the scholar did not enumerate how to effectively manage the knowledge transfer between partners [6]. The purpose of Offong et al.'s research is to investigate whether individuals' attitudes toward the use of corporate social media can affect tacit knowledge sharing and work performance. Through his experiments, he found that the use of various software has a great relationship with trust. However, this will not affect knowledge transfer. He found that trust can be promoted through online participation among employees. However, the scholar did not design the reference data in the experiment, which made the experiment lose its reliability [7]. Gou et al. found that as the dynamics of the external environment of the enterprise continue to increase, the support of information systems for organizational agility has become more and more important. He found that effective knowledge transfer is the core of system implementation. His research results show that by exploring knowledge transfer issues in new environments, the implementation methods of agile information systems can be enriched. However, the scholar did not provide corresponding data support for the conclusion, making the experiment not very real and lacking persuasiveness [8].

## 3. Basic Concepts of Virtual Enterprise and Cognitive Computing

Driven by the wave of global marketization, the extensive use of information technology has enabled corporate organizations to break through the tangible boundary constraints in the process of forming core competitiveness. The virtual organization has gradually become a wide range of cooperation modes in enterprise innovation and development. With the development of science and technology, virtual enterprises have gradually become the main body of market competition in recent years. A virtual enterprise is a temporary network formed through the connection of information technology, infrastructure, and shared business processes to meet the needs of a specific market [9]. The development and application of virtual enterprises are shown in Figure 1.

As shown in Figure 1, because the structural analysis method is an effective modeling tool for solving complex open systems, this method is generally used to solve the multilevel network structure of virtual enterprise information management [10]. The structural analysis method is a scientific analysis method to understand the overall characteristics of things by analyzing and establishing the connection methods between the internal components of things. Any objective thing is a whole with a certain structure, and structural analysis has become the basic method for people to understand things.

Based on the considerations, based on the theoretical research of the virtual enterprise information management model, this study locally develops the virtual enterprise information management system so that the enterprise can quickly adapt to the fierce competition on a global scale [11]. The development process of virtual enterprises is shown in Figure 2.

As shown in Figure 2, the multilevel network structure of a virtual enterprise determines that the theoretical research of its information management model must have a certain level of hierarchy [12]. The multilevel interconnection network is composed of a large number of basic switching modules connected to each other according to a specific topological structure, forming a larger-scale switching network capable of information exchange. The structural analysis method provides an effective way to discuss the information processing, coordination, and control of the virtual enterprise and at the same time improves the agility of the enterprise to adapt to the large-scale global market and fierce competition.

This study investigates the development trend of virtual enterprises from 2015 to 2019, as shown in Table 1.

As shown in Table 1, in 2015, the number of virtual enterprises was 5,678, with a growth rate of 13%. In 2018, the number of virtual enterprises was 10,250, with an increase of 4,572, and with a growth rate of 36%. The development of virtual enterprises from 2015 to 2019 is very rapid. The “virtual enterprise” defined in this study is a virtual enterprise that adapts to the changes in the environment and summarizes the independent enterprises with core functions in the various links of the value chain. A virtual enterprise is centered on knowledge, projects, products, or services. It has no independent enterprise form, but it can realize specific enterprise functions [13]. The basic structure of a virtual enterprise is shown in Figure 3.

As shown in Figure 3, the core layer of a virtual enterprise is composed of one or more enterprises, and the core members are closely connected and relatively stable. The overall construction of a virtual enterprise is mainly composed of core team members, which is the best decision-making and adjustment mechanism for a virtual enterprise.

The virtual enterprise cross-organizational interface knowledge management technology model is divided into knowledge alliance layer, knowledge screening layer, knowledge content layer, and knowledge application [14], as shown in Figure 4.

As shown in Figure 4, through contract constraints, virtual enterprise knowledge alliances are formed. This layer is mainly to provide support and guarantee for virtual enterprise knowledge management.

Cognitive computing is an important part of artificial intelligence and one of the important fields of the core technology of cognitive science. It is a computer system that simulates the cognitive process of the human brain [15]. Cognitive computing represents a new computing model. It includes a number of technologies in the fields of information analysis, natural language processing, machine learning, etc., which help decision-makers to gain extraordinary insights into a large amount of unstructured data [16], as shown in Figure 5.

As shown in Figure 5, cognition is the human's cognitive activity of the objective world. The human brain receives information input from external sensory organs, through the analysis and processing of the brain, it rises to the inherent spiritual activity of human beings, and then, it dominates the brain [17]. The essence of cognitive computing is to allow computers to imitate human cognitive mechanisms.

## 4. Principal Component Analysis Algorithm and Cloud Model Algorithm Based on Cognitive Computing

### 4.1. Principal Component Analysis Algorithm Based on Cognitive Computing

Although the research on cognitive computing is active, it is still in the early stage of research and will be an important topic for the development of artificial intelligence in the future [18], as shown in Figure 6.

As shown in Figure 6, cognitive computing is derived from artificial intelligence that simulates the human brain system and has a huge impact on people's lives [19].

The principal component analysis is a statistical method. Through orthogonal transformation, a group of variables that may be correlated is transformed into a group of linearly uncorrelated variables. The transformed group of variables is called the principal component. The main idea of the principal component analysis method is to reduce the dimensionality of the sampling space as much as possible under the premise of ensuring sufficient information and to reduce the dispersion of maximizing sampling to minimize the mean square error of reconstruction. The following introduces the principal component analysis method defined by maximizing the sample variance of the projection space [20]. Given sample set *a*_*i*_ ∈ *R*^*m*^(1,2,…, *n*) of *n* samples, let *h* ∈ *R*^*m*^ be the orthogonal projection direction, as in

(1) $$\begin{array}{c} \left\|h\right\|=h^{T}h=1. \end{array}$$

The projection of sample *a*_*i*_ to *h* is

(2) $$\begin{array}{c} b_{i}=h^{T}a_{i}. \end{array}$$

Then, the sample variance in the projection space is

(3) $$\begin{array}{c} S^{2}=\frac{1}{n-1}\sum_{i=1}^{n}\left(b_{i}-b\right), \end{array}$$

where *a* is the mean value of the sample in the projection space. According to the principle of principal component analysis, maximizing the sample variance in the projection space is

(4) $$\begin{array}{c} \max h=\frac{1}{n-1}\sum_{i=1}^{n}\left(a_{i}-a\right){\left(a_{i}-a\right)}^{T}. \end{array}$$

Then, the problem is transformed into a conditional extreme optimization problem *f*(*h*, *λ*), which is

(5) $$\begin{array}{c} f\left(h,\lambda \right)=h^{T}Ch+\lambda \left(1-h^{T}h\right). \end{array}$$

Given sample set *a*_*i*_ ∈ *R*^*m*^(1,2,…, *n*) of *n* samples, let matrix *A*=(*a*_1_, *a*_2_,…, *a*_*n*_) ∈ *R*^*m*×*n*^. The sample mean is

(6) $$\begin{array}{c} A=\frac{1}{n}\sum_{i=1}^{n}a_{i}. \end{array}$$

Among them, the sample projection subspace *H*=(*h*_1_, *h*_2_,…, *h*_*n*_) ∈ *R*^*m*×*n*−1^ and eigenvalue is *λ*_1_, *λ*_2_,…, *λ*_*n*−1_. The eigenvectors corresponding to the first *k*(*k* ≺ *n* − 1) eigenvalues are selected to form H, and the test sample *a* ∈ *R*^*m*^ is projected. The sample matrix is normalized by the mean to obtain *A*=(*a*_1_, *a*_2_,…, *a*_*n*_), where the sample covariance matrix is

(7) $$\begin{array}{c} C=\frac{1}{n-1}AA^{T}. \end{array}$$

Projection *a* is obtained as

(8) $$\begin{array}{c} a=H_{k}^{T}a^{i}\left(h\in R^{n-1}\right). \end{array}$$

The basis of the selected *k* feature vectors can retain most of the original information. *H*_*k*_^*T*^ is the principal component of the original sample set.

General self-efficacy is the degree of self-confidence of the individual's ability and resources needed to achieve goals, which has a direct impact on the perception of efficacy in a specific field. Perceptual autonomous learning is based on the learning of growth memory. When input perception can search for related actions in long-term memory, the actions are directly output for the next step of learning [21], as shown in Figure 7.

As shown in Figure 7, driven by working memory, the perceptual model continuously explores and learns new knowledge, and such new knowledge is the new perceptual action mapping. When input perception cannot find a related action in long-term memory, it is considered as a new perception and its action meaning is given. The associated action vector is extended to the perceptual vector to form the perceptual action mapping vector for long-term memory learning [22].

Recall algorithm is an important method for learning data streams with concept drift. Aiming at the defects of traditional integrated data stream mining, human memory and forgetting mechanisms are introduced into data stream mining. When there is an action corresponding to the input perception in the network, the recall algorithm is used to find the corresponding action vector output. The perceptual action mapping recall algorithm is as in

(9) $$\begin{array}{c} d_{k↔i}=\frac{\left\|G-W_{i}^{a}\right\|}{\sqrt{m}}. \end{array}$$

By inputting the perception vector K, the average distance between K and other nodes is *d*_*k*↔*i*_.

Perception mapping *ξ*=*H*_1_^*T*^*a*_*t*_, finds the corresponding action output of the perception and calculates the average distance between *ξ* and other nodes as

(10) $$\begin{array}{c} d_{k↔i}=\left\{\begin{array}{c} \frac{\left\|\xi -W_{i}^{a}\right\|}{\sqrt{m}},\\ \frac{\left\|\xi -W_{i}^{G}\right\|}{\sqrt{m}}. \end{array}\right. \end{array}$$

### 4.2. Cloud Model Algorithm

Cognition is a kind of mental activity. It is the process of information processing by the human brain. It includes perception, memory, judgment, and so on. It is the process of mankind's in-depth understanding of the objective world, and it is also a process of understanding from the outside to the inside. With the development of artificial intelligence technology, artificial intelligence technology that simulates the information processing process of the human brain has become a hot spot. Cognitive computing based on the cloud model is one of the important theories in this technology.

The cloud model can simulate human thinking and flexibly divide the attribute space and complete the conversion from quantitative values to qualitative concepts. At the same time, the overlap between adjacent attribute values or languages is allowed. This division makes the discovered knowledge robust. The cloud model is a model for studying the connotation of the uncertainty concept in uncertainty artificial intelligence. Its research object is the ambiguity and randomness of the attributes of objective things. Traditional cognitive computing and cloud-based cognitive computing are shown in Figure 8.

As shown in Figure 8, through the study of different transformation methods of the cloud model, the various stages of human cognition are studied to realize the description of the entire human cognition process and then establish a computing model with the characteristics of human thinking.

Suppose *U* is a quantitative domain represented by an accurate numerical value, *C* is a qualitative concept described by numbers on *H*, if the quantitative value is *Y* ∈ *H*, and *Y* is a random reality of the qualitative concept *C*. The certainty *μ* ∈ [0,1] of *Y* to *C* is a stable random number, as shown in

(11) $$\begin{array}{c} \left\{\begin{array}{cc} \mu : & H⟶\left[0,1\right],\\ \forall_{Y}\in H, & Y\;\mapsto \;\mu \left(Y\right). \end{array}\right. \end{array}$$

Each *Y* is called a cloud drop in the universe of discourse.

The cloud model is a mathematical model that focuses on the connection between randomness and ambiguity. In practical applications, the contribution of Yundi alone to the concept is small. Only a large number of cloud drops work together to form the connotation of the concept.

*Y* satisfies *Y*=*R*(*E*_*Y*_ *|* *Y*), where the certainty of *Y* to *C* satisfies

(12) $$\begin{array}{c} H\left(Y\right)=e^{-\left({\left(y-E_{y}\right)}^{2}/2y^{2}\right)}. \end{array}$$

*Y*=*R*_*n*_(*E*_*n*_, *H*_*e*_) represents a normal random number with *E*_*n*_ as the expectation and *H*_*e*_ as the standard deviation.

For the contribution of the second-order normal cloud drop, the contribution of the cloud drop to the qualitative concept can be obtained by formula (12), that is,

(13) $$\begin{array}{c} \Delta C\approx \frac{\mu_{A}\cdot \Delta Y}{\sqrt{2\pi }E_{n}}. \end{array}$$

Among them, Δ*Y* is the cloud drop group, and Δ*C* is the contribution of Δ*Y* to the qualitative concept. Formula (13) can be used to deduce all cloud drops in the universe of discourse, and its total contribution to the qualitative concept is 1.

Among all the elements, the elements with the highest contribution rate are almost all within the range of the backbone elements and basic elements, and the certainty of the elements corresponding to the region is relatively high, which also reflects the characteristics of human cognition. Mankind sums up a large amount of history and derives regular knowledge from it.

The cloud model algorithm uses normal random numbers to generate cloud drops, and the process of generating cloud drops conforms to probability theory. The generation of one cloud drop is the condition for another generation, and the second-order normal cloud drop is

(14) $$\begin{array}{c} Y_{i}=R_{N}\left(E_{Y},\left|Y_{i}\right|\right). \end{array}$$

And because of *Y*_*i*_=*R*_*N*_(*E*_*Y*_, *H*_*e*_), the probability density function of *Y* is

(15) $$\begin{array}{c} f_{y}\left(y\right)=\frac{e^{-\left({\left(y-E_{N}\right)}^{2}/2H_{e}^{2}\right)}}{\sqrt{2\pi }\left|y\right|}. \end{array}$$

When the random variable *Y*=*y* is a fixed value, because of *Y*=*R*_*N*_(*E*_*Y*_|*Y*|), the probability density function of *Y* is

(16) $$\begin{array}{c} f_{x/y}\left(x\;|\;y\right)=f_{x/y}\left(x\;|\;y=y\right)f_{Y}\left(y\right). \end{array}$$

It can be seen from formula (16) that the certainty of cloud drops depends on the changes in *X* and *Y*. The random variable *H*(*Y*) of certainty is

(17) $$\begin{array}{c} f_{z/y}\left(z\;|\;Y=y\right)=\frac{1}{\sqrt{-\pi \text{inz}}},\;0\;≺\;z\;≺\;1. \end{array}$$

When *X*=*x* is a constant value, the density function is

(18) $$\begin{array}{c} f_{Z/X}\left(z\;|\;Y=X\right)=\frac{\left|X-E_{X}\right|}{4z\sqrt{\pi \text{inz}}H_{e}}{\left(-\text{inz}\right)}^{-1},\;0\;≺\;z\;≺\;1. \end{array}$$

It can be seen from formula (18) that the probability density function is related to the values of *E*_*n*_ and *E*_*Y*_. For a cloud drop, the degree of certainty is not a certain value, which is caused by the uncertainty and difference in the degree of human awareness of the concept in the activity of concept cognition. Therefore, the degree of certainty reflects the ambiguity and randomness of human cognition, as shown in

(19) $$\begin{array}{c} f_{Z}\left(Z\right)=\frac{1}{\sqrt{-\pi \text{inz}}},\;0\;≺\;z\;≺\;1. \end{array}$$

$\sqrt{-\pi \text{inz}}$ The certainty of the elements must appear a unified state as a whole. This is the commonplace between the cloud model and the human cognition process, and it is consistent with the law of human cognition.

In this study, we also apply a certain degree of reverse cloud conversion algorithm, that is, using the certainty of the sample and the sample itself, and the three parameters of the second-order normal cloud are obtained in reverse. Assuming that the sample *Y* and its certainty are *Y*_*i*_, the estimator *E*_*Y*_ is the mean value of the sample. Here,

(20) $$\begin{array}{c} E_{Y}=Y_{i}=\frac{1}{n}\sum_{i}^{n}Y_{i}. \end{array}$$

The calculation basis of the inverse cloud transformation algorithm without certainty is the statistical characteristics of the elements. The digital feature estimator in the normal cloud model is obtained through the statistics of cloud drops, so it is a more practical calculation method.

## 5. Experiment and Analysis of the Influencing Factors and Measures of Virtual Enterprise Knowledge Transfer

### 5.1. Experiment and Analysis of Factors Affecting Knowledge Transfer of Virtual Enterprises

The emergence of virtual enterprise has broken the stability of the traditional enterprise industry boundary, and it is an open complex dynamic system. The impact of virtual enterprises on various regions of China is shown in Table 2.

It can be seen from Table 2 that this study separately investigated virtual enterprises in the eastern, central, southern, northern, and northwestern regions. A survey was also conducted on the local employment rate of virtual enterprises, the exchanges between various regions, the development of enterprises, and their contribution to regional funds. After investigation, it is found that virtual enterprises have enabled the employment rate in the east to reach 27%, the flow rate between the local and various regions has reached 35%, and the capital contribution has reached 456.7 million U.S. dollars. The employment rate in central China has reached 29%; virtual enterprises have enabled the employment rate in central China to reach 29%, making the flow rate between the local and various regions reach 37%, and the capital contribution has reached 675.31 million U.S. dollars. Virtual enterprises have enabled the employment rate in the northwest region to reach 30%, the flow rate between the local and various regions has reached 36%, and the capital contribution has reached 978.06 million U.S. dollars. It has made the greatest contribution to the northwest region. It can be seen that the development of virtual enterprises has brought a huge impact on people.

Virtual enterprise knowledge transfer is the basis and process for virtual enterprise members to learn knowledge and abilities from each other and strengthen their own abilities. However, this kind of knowledge transfer will be affected by many factors. This study analyzes three aspects: knowledge factor, virtual enterprise member factor, and the virtual enterprise itself. In this study, the influence of knowledge factors is first investigated, as shown in Figure 9.

As shown in Figure 9, the influence of knowledge factors is mainly explicit knowledge and tacit knowledge. The efficiency of explicit knowledge has risen from about 7% at the beginning to about 16% afterward. In the process of knowledge transfer, the transfer of explicit knowledge is relatively simple and can be immediately used after transfer; tacit knowledge is more difficult to identify and difficult to communicate. At the same time, it takes time to digest the knowledge after transmission.

The member factors of the virtual enterprise are divided into knowledge transfer party and knowledge receiver. In this study, we conduct separate investigations on the knowledge transfer party and knowledge receiver of the virtual enterprise member factors, and each selects 5 representatives to score for the investigation, as shown in Tables 3 and 4.

As shown in Table 3, the influencing factors of the knowledge transfer party on the knowledge transfer include interest factors, the knowledge transfer party's willingness to transfer, the reliability of the knowledge transfer party, the communication ability of the knowledge transfer party, and the coding ability. Among them, 5 representatives gave the highest score of 8.3 points for the benefit factor, and the lowest score was 7.8 points. On average, these factors scored the highest, so the benefit factor is the most critical factor.

Benefit factor: knowledge as a resource requires time, energy, wealth, and other costs to obtain. The parties involved in knowledge transfer often worry that they will not get appropriate benefits after the knowledge transfer or are unwilling to provide time to support the knowledge transfer.

The transfer willingness and reliability of the knowledge transfer party: when the knowledge transfer is related to the source of core knowledge and core competence, the knowledge transfer party is unwilling to transfer the knowledge. As if the core knowledge is transferred, the company's advantages or competitiveness may be reduced or even lost. On the contrary, if the transferred knowledge does not belong to the core knowledge, it will not affect the competitiveness of the enterprise, and the knowledge transfer party will be willing to transfer the knowledge. When the reliability of the enterprise's knowledge is not verified, the knowledge transfer will not be accepted by the recipient, so the knowledge transfer is also very difficult.

The communication ability of the knowledge transfer party: if the knowledge transfer party has good communication skills and is good at dealing with people, then the transfer of knowledge will smoothly proceed. If the communication ability of the knowledge transfer party is poor, others will not be interested in knowing the knowledge of the enterprise. At this time, the receiver will receive very little knowledge.

As shown in Table 4, the influencing factors of knowledge beneficiaries in knowledge dissemination include the learning intention of the knowledge beneficiaries, the absorptive capacity of the knowledge beneficiaries, the communication ability of the knowledge beneficiaries, and the initiative of the knowledge beneficiaries.

The learning intention of the knowledge receiver: the learning intention of the knowledge receiver will directly affect the knowledge transfer. As if the learning intention of the knowledge receiver is stronger, he will actively learn the transferred knowledge, which will improve the efficiency of knowledge transfer. On the contrary, if the learning intention of the knowledge receiver is poor, his initiative to learn the transferred knowledge will also become poor, resulting in slower knowledge acceptance and lower efficiency.

Absorptive capacity of the knowledge receiver: the ability of the knowledge receiver to digest, transform, and apply the transferred knowledge also affects the learning effect of the knowledge transferrer in the virtual enterprise. In short, the higher the absorptive capacity of the knowledge receiver, the more chance it will convert the knowledge transferred by the knowledge transfer party into the enterprise's own knowledge.

This study investigates the influence of virtual enterprise A and virtual enterprise B's own factors on knowledge transfer, as shown in Figure 10.

As shown in Figure 10, the virtual enterprise's own factors include good learning habits, trust between members, and the enterprise environment. The learning habits of virtual enterprise A are better than those of virtual enterprise B, so the knowledge transfer efficiency of virtual enterprise A is also higher than that of virtual enterprise B. The trust among members of virtual enterprise A is also stronger than that of virtual enterprise B, which leads to a higher knowledge transfer efficiency of virtual enterprise A than virtual enterprise B. The environment of the virtual enterprise A is also better than that of the virtual enterprise B. Combining the above discussion, we can see that good study habits, a high degree of trust between members, and a good corporate environment will increase the efficiency of knowledge transfer.

### 5.2. Measures to Promote Knowledge Transfer in Virtual Enterprises

#### 5.2.1. Establishing a Transparent Cooperative Relationship

In order to enhance the willingness of virtual enterprises to transfer knowledge, member companies should strive to establish a transparent cooperative relationship and adopt an open and honest attitude to design a transparent mechanism that is conducive to knowledge sharing, transfer, and absorption. To stimulate the enthusiasm of member companies to share and transfer knowledge, multifaceted display of the benefits of knowledge transfer in the process of project cooperation is needed.

#### 5.2.2. Knowledge and Technical Reserves of Corporate Members

The knowledge and technical reserves of enterprise members are the key to the knowledge transfer of virtual enterprises, and the effective ways and means of knowledge accumulation are mainly through the construction of learning enterprise organizations. Aiming at the characteristics of virtual enterprise knowledge learning, constructing a learning virtual organization within the scope of the virtual enterprise is an important guarantee for virtual enterprise knowledge transfer.

#### 5.2.3. Creating a Good Knowledge Transfer Environment

The purpose of virtual enterprise knowledge transfer is to acquire the tacit knowledge of partners through learning and improve its own innovation ability. In an effective learning organization, creating an excellent mutual learning environment and encouraging continuous learning and communication between employees and the company are a prerequisite for effective learning and knowledge accumulation.

#### 5.2.4. Choosing a Knowledge Transfer Management Model That Fits the Type of Virtual Enterprise

Different types of virtual enterprises have different purposes and requirements for knowledge transfer, and the modes of knowledge transfer management are also different. Therefore, the choice of knowledge transfer management mode is the primary task of virtual enterprise knowledge transfer management, which directly affects the implementation effect of virtual enterprise knowledge transfer management.

## 6. Discussion

This study analyzes how to conduct research on virtual enterprise knowledge transfer and knowledge management based on structured cognitive computing. The related concepts of virtual enterprise and cognitive computing are expounded, and the principal component analysis algorithm and cloud model algorithm based on cognitive computing are studied. It analyzes the virtual enterprise, explores the method of cognitive computing research, and the experiment and analysis of various algorithms to understand the importance of cognitive computing and the analysis of knowledge transfer in the virtual enterprise. Finally, the analysis is carried out by taking cognitive computing integrated into the knowledge transfer analysis of virtual enterprises as an example.

This study also makes reasonable use of the principal component analysis algorithm and cloud model algorithm based on cognitive computing. As the application scope of the two algorithms becomes larger and larger, their importance also increases. Many scholars have begun to apply principal component analysis algorithms and cloud model algorithms to all aspects of life. According to these two algorithms, based on the principal component analysis algorithm and the cloud model algorithm, it is very meaningful to study the knowledge transfer of virtual enterprises.

Through experimental analysis, this study knows that with the development of virtual enterprises, the role of knowledge transfer is also increasing. There are many factors that affect knowledge transfer. The experiment in this study proposes specific measures for various factors, so as to promote the healthy and stable development of virtual enterprise knowledge transfer.

## 7. Conclusions

This study explains the importance of virtual enterprises to the development of contemporary society, leading to the importance of knowledge transfer to virtual enterprises. How to promote the development of virtual enterprises by knowledge transfer can be analyzed through structured cognitive computing. This study provides a theoretical overview of virtual enterprises and cognitive computing. In the method part, based on cognitive computing, the principal component analysis algorithm and the cloud model algorithm are described in detail, and the reason for using the cloud model algorithm to analyze knowledge transfer and management is explained. The experimental part found that the factors affecting the normal development of knowledge transfer include knowledge factors, virtual enterprise member factors, and virtual enterprise own factors. The knowledge factor also includes explicit knowledge and tacit knowledge, both of which have different effects on knowledge transfer. Virtual enterprise member factors are divided into knowledge transfer parties and knowledge receivers. The initiative and communication skills between the two parties directly affect whether the knowledge can be smoothly transferred. If we want to make the transfer of knowledge between virtual enterprises normally and healthily proceed, we must take measures against these factors. Enterprises should trust each other, actively transfer, and accept knowledge, and enterprises should also actively create a good transfer environment. In conclusion, the smooth progress of knowledge transfer will affect the development of virtual enterprises.

## Figures and Tables

**Figure 1:** Development and application of virtual enterprises.

**Figure 2:** The development history of virtual enterprises.

**Figure 3:** The basic structure of a virtual enterprise.

**Figure 4:** Virtual enterprise knowledge management system.

**Figure 5:** Basic structure of cognitive computing.

**Figure 6:** Cognitive computing process.

**Figure 7:** Perceived autonomous learning.

**Figure 8:** (a) Traditional cognitive computing. (b) Cloud model-based cognitive computing.

**Figure 9:** Influencing factors of knowledge factors.

**Figure 10:** The influence of (a) virtual enterprise A and (b) virtual enterprise B's own factors on knowledge transfer.

**Table 1:** The development trend of virtual enterprises from 2015 to 2019.

Year	Quantity	Growth rate (%)	Funds
2015	5678	13	345622
2016	6784	18	543536
2017	7923	21	657854
2018	8702	25	789532
2019	10250	36	906753

**Table 2:** The impact of virtual enterprises on various regions of China.

Area	Employment rate (%)	Flow rate (%)	Enterprise development rate (%)	Fund contribution
East	27	35	56	$45673
Central	29	37	58	$67531
South	25	36	55	$77392
North	24	34	57	$89764
Northwest	30	36	53	$98706

**Table 3:** Influencing factors of knowledge transfer party on knowledge transfer.

	1	2	3	4	5
Benefit factor	7.8	7.9	8.3	8.2	8.0
Willingness to transfer	6.4	6.8	6.7	6.6	6.7
Transfer reliability	6.3	6.4	6.8	6.1	5.8
Communication and coding skills	5.7	5.9	5.3	5.5	5.8

**Table 4:** Influencing factors of knowledge receivers on knowledge transfer.

	1	2	3	4	5
Learning intention	8.3	7.4	7.5	8.1	7.4
Absorptive capacity	8.1	7.5	6.4	7.5	7.3
Communication	7.5	7.8	6.9	6.7	7.7
Initiative	7.6	7.6	6.3	7.0	7.5

## Data Availability

The authors do not have permission to share data from the data provider.
